# Rib Fracture Detection with Dual-Attention Enhanced U-Net

**DOI:** 10.1155/2022/8945423

**Published:** 2022-08-18

**Authors:** Zhengyin Zhou, Zhihui Fu, Juncheng Jia, Jun Lv

**Affiliations:** ^1^School of Computer Science and Technology, Soochow University, Suzhou 215006, China; ^2^Department of Radiology, Suzhou TCM Hospital Affiliated to Nanjing University of Chinese Medicine, Suzhou 215000, China; ^3^School of Computer and Control Engineering, Yantai University, Yantai 264005, China

## Abstract

Rib fractures are common injuries caused by chest trauma, which may cause serious consequences. It is essential to diagnose rib fractures accurately. Low-dose thoracic computed tomography (CT) is commonly used for rib fracture diagnosis, and convolutional neural network- (CNN-) based methods have assisted doctors in rib fracture diagnosis in recent years. However, due to the lack of rib fracture data and the irregular, various shape of rib fractures, it is difficult for CNN-based methods to extract rib fracture features. As a result, they cannot achieve satisfying results in terms of accuracy and sensitivity in detecting rib fractures. Inspired by the attention mechanism, we proposed the CFSG U-Net for rib fracture detection. The CSFG U-Net uses the U-Net architecture and is enhanced by a dual-attention module, including a channel-wise fusion attention module (CFAM) and a spatial-wise group attention module (SGAM). CFAM uses the channel attention mechanism to reweight the feature map along the channel dimension and refine the U-Net's skip connections. SGAM uses the group technique to generate spatial attention to adjust feature maps in the spatial dimension, which allows the spatial attention module to capture more fine-grained semantic information. To evaluate the effectiveness of our proposed methods, we established a rib fracture dataset in our research. The experimental results on our dataset show that the maximum sensitivity of our proposed method is 89.58%, and the average FROC score is 81.28%, which outperforms the existing rib fracture detection methods and attention modules.

## 1. Introduction

Rib fractures are associated with significant morbidity and are detected in at least 10% of all injured patients [1], with patients frequently requiring admission to the intensive care unit (ICU) and mortality rates as high as 33% [2]. To avoid serious consequences, accurate detection of rib fractures is important. Low-dose thoracic computed tomography (CT) scans are commonly used in the assessment and auxiliary diagnosis of rib fractures [3, 4], but missed diagnoses are common. Studies have shown that the sensitivity of diagnosis of rib fractures is only about 60% on initial chest CT evaluations [5], and missed diagnosis may cause severe medical accidents. Moreover, it is time-consuming for radiologists to find and locate rib fractures in numerous CT slices.

Artificial intelligence (AI) has recently made remarkable progress. It is widely used in medical data analysis, such as detection of diabetic retinopathy [6], classification of neonates cry [7], and analysis of electroencephalogram (EEG) signals [8]. The detection of rib fracture can be regarded as a computer vision task. Deep convolutional neural networks (CNNs) are used to extract the features hard to find by human beings and achieve the state-of-the-art performance in many computer vision tasks [9–13]. As for computer-aided diagnosis, CNNs are widely used for segmentation, detection, and classification of lesions in medical images, such as lung nodule detection and classification [14–16], brain tumor segmentation [17–19], breast cancer detection and classification [20–22], which demonstrate their extraordinary ability to outperform medical professionals.

Motivated by the successful application of CNNs in computer-aided diagnosis, several initial attempts have been made to design rib fracture detection algorithms based on CNNs in recent years. For instance, Chen et al. [23] presented a spatial coherence-based rib fracture detection method to detect rib fractures. They first gave a novel feature extraction method to extract the rib regions from CT slices. Then, for each rib region, they applied a spatial coherence convolutional neural network to recognize rib fractures. Zhou et al. [24] used Faster R-CNN [25], a two-stage region-based object detection model, to locate and classify rib fractures in 2D CT slices. Jin et al. [26] proposed a 3D CNN network called FracNet, based on U-Net [27], to segment the rib fracture region from a single cut patch. Then, they applied a sliding window mechanism for the whole 3D CT volume to detect rib fractures. Meng et al. [28] proposed a fully automated rib fracture detection pipeline consisting of five stages: rib segmentation, vertebra detection, rib labeling, rib fracture detection, and rib fracture classification. In the rib fracture detection stage, the proposed model VRB-net was used to locate the fracture and output the probability map, which is based on the V-Net structure and includes a ResNet module (R-module) and a bottleneck ResNet module (B-module). These works use 2D or 3D CNNs to detect rib fractures and have achieved good results. But there is still research space of improving the CNN network's ability to get a better result in rib fracture detection tasks. There are still some problems with rib fracture detection using CNN networks. On the one hand, it is challenging to collect rib fracture data due to obstacles such as privacy ethics and data labeling cost, which lead to limited training data. On the other hand, some of the rib fracture regions are not apparent compared with the normal rib regions. With the narrow shape of ribs and various irregular fracture structures, rib fractures can be easily confused with normal ribs in CT images and misdiagnosed. These issues limit the performance of CNN models.  Table 1 lists the relevant works and the challenges they face.

The attention mechanism has been widely studied recently in various AI areas. The idea of the attention mechanism is to focus on essential information and quickly obtain the most effective information, which can help the CNN network learn more fine-grained information from the samples to improve the feature extraction ability. Inspired by the attention mechanism, we proposed a U-Net-based rib fracture detection algorithm for automatic and accurate rib fracture detection called CFSG U-Net. To improve the detection performance in our algorithm, we proposed a dual-attention mechanism to help the network learn rib fracture features from limited data, which includes a channel-wise fusion attention module (CFAM) and a spatial-wise group attention module (SGAM). CFAM focuses on the channel relationship in CNNs, and adaptively redistributes the weights of features along the channel dimension. Besides, we also use CFAM to refine the U-Net's skip connections. The study has shown a semantic gap between low-level and high-level features merged in U-Net's long skip connections [29, 30], which hurts the network's performance. CFAM is used to adjust these two sets of features before convolutional blocks merge them to help them fuse effectively. SGAM focuses on spatial information and adjusts the weights along the spatial dimension. Commonly spatial attention in [31, 32] uses average-pooling or max-pooling to aggregate channel-wise information, which may lose fine-grained information and cannot fully characterize the various semantic information of the feature map. To solve this problem, we divide feature maps into several groups. Each group generates channel-wise statistics individually to learn spatial attention maps, allowing spatial attention to capturing more fine-grained semantic information.

To verify the performance of our proposed method, we established a dataset of rib fractures from the local hospital's patients, including 3134 rib fracture annotations for 818 CT images.

The contributions of this paper are summarized as follows:

- We propose the CFSG U-Net for automatic rib fracture detection, which is enhanced by our proposed novel dual-attention mechanism including CFAM and SGAM
- We established a rib fracture dataset, including 3134 rib fracture annotations for 818 CT images
- Our proposed method achieves a sensitivity of 89.58%, and the average FROC score is 81.28% on our dataset, which outperforms the state-of-the-art methods.

## 2. Materials and Methods

### 2.1. Ethics

All procedures involving human participants in this retrospective study were approved by the ethics committee of Suzhou TCM Hospital Affiliated to the Nanjing University of Chinese Medicine. The requirement for informed consent was waived according to the ethical standards of the institutional review board.

### 2.2. Materials

A total of 818 patients participated in this study. We collected 818 CT images of patients with chest trauma between March 2017 to April 2019 from the hospital's picture archiving and communication systems (PACS). There are 511 male and 307 female patients, with an average age of 57. All CT scans were acquired from a CT machine with a voltage of 270 kV and a current of 200-300 mA, stored in digital imaging and communications in medicine (DICOM) format. The scan thickness was 1.25-5 mm.

Three experienced musculoskeletal radiologists completed the annotation of CT images. Two have more than five years of experience in musculoskeletal CT imaging diagnosis, and the senior one has more than ten years of experience. Firstly, all CT images were checked by two junior doctors, combined with the perspectives of the coronal, sagittal, and horizontal planes, to find out and locate the rib fractures and mark them with 3D masks. The results of the initial annotation were reviewed by the senior radiologist and confirmed the final ground truth. All CT images were annotated by ITK-SNAP [33], and the labels were exported in neuroimaging informatics technology initiative (NIFTI) format. Finally, 3134 annotations were acquired. An example of the annotation can be seen in Figure 1.

The dataset was randomly divided into three parts, including the training set, validation set, and test set with a ratio of 7 : 1 : 2. We trained the model on the training set and adjusted the hyperparameters on the validation set to obtain the model with the best performance. Finally, we tested the model's actual performance on the test set.

### 2.3. Data Preprocessing

In addition to the bone region, chest CT contains information about other tissues. Such redundant information may negatively impact prediction accuracy and detection speed. Removing these redundant tissues is an intuitive way to avoid such negative impacts. For this purpose, we use a series of morphological operations to extract the bone regions in the CT image and then normalize the results to obtain the final input data for the neural network. The overall procedure is illustrated in Figure 2.

The original image is shown in Figure 2(a). If we extract the largest connected components directly after binarizing the image using a certain threshold to obtain the bone region, some ribs may be lost, especially for the eleventh and twelfth ribs. Therefore, we remove small connected components and apply dilation operations before extracting the largest connected components.

First, we select the threshold of 180 *HU* to binarize the image to capture the high-intensity bone region (Figure 2(b)). After that, the connected components include bone regions and other redundant tissues and noise. If we make a dilation operation immediately, these distracting components will be mixed with the bone areas. Therefore, before the dilation operation, we remove the connected components smaller than 4000 mm^3^ in volume (Figure 2(c)). The surrounding areas of bone tissues, including cortical and bone marrow, are important for diagnosing rib fractures, but the mask cannot completely cover these areas after binarization. Therefore, we make a morphological dilation operation to expand the regions and fill small holes (Figure 2(d)). After all the above operations, we extract the largest connected components to obtain the bone region mask we need (Figure 2(e)). Finally, we multiply the bone region mask with the original image, all parts within the mask retain the original information, while everything outside the mask is filled with -300 *HU*. The extracted bone region can be seen in Figure 2(f).

To make the bone clear, we adjust the CT image to the bone window, the window width is 1200, and the window level is 300. Finally, we use min-max normalization to transform the data to the range [0, 1]. The formula for min-max normalization is as follows:

(1) $$\begin{array}{c} x^{\prime }=\frac{x-\min\left(x\right)}{\max\left(x\right)-\min\left(x\right)}. \end{array}$$

The final output of preprocessing can be seen in Figures 2(g) and 2(h).

### 2.4. Proposed Neural Network Structure

Our proposed CFSG U-Net uses the encoder-decoder structure based on U-Net, a widely used architecture for medical image segmentation. The detailed design of our proposed network is shown in Figure 3.

In the encoder path, CSFG U-Net gradually downsamples and doubles the number of channels. In contrast, in the decoder path, the resolution is restored step by step with transpose convolution, and the number of channels is reduced by convolution; skip connections are used to introduce the fine-grained information of low-level features to help the feature map restore the resolution.

The encoder block includes convolutional layers, batch normalization, and ReLU activation function. Moreover, the residual connections proposed by He et al. [34] are introduced to extract more accurate rib fracture features. Recent work [35, 36] has shown that convolution may lose information, while residual connections can help deliver contextual information, improve segmentation accuracy, and accelerate the convergence speed. After that, max-pooling layers are used to downsample the feature maps.

In the decoder block, we propose a channel-wise fusion attention module (CFAM) to reweight the feature map along the channel dimension and refine the U-Net's skip connections. The CFAM considers the interchannel relationship between low-level and high-level features and uses the attention mechanism to adjust these two sets of features before fusing them. Inspired by the group technique, we introduce a spatial-wise group attention module (SGAM), which can learn spatial attention maps in a group manner. The attention map of each group attends to a specific semantic feature, which can reserve more spatial structural information and help the spatial attention module capture more fine-grained semantic information.

In the decoder block, the low-level features from the encoder path and the high-level features from the decoder path are refined by CFAM and then fused by a convolution block. After that, the SGAM is used to refine the features spatially. At last, a convolution block is used to learn features and help the network adapt to the attention mechanism. Residual connection is also used to fine-tune the features.

### 2.5. Channel-Wise Fusion Attention Module

The overall architecture of CFAM is illustrated in Figure 4(a). CFAM is a channel attention module that strengthens useful feature responses and suppresses unimportant feature responses by adjusting the relationship along the channel dimension. But unlike the classic channel attention like SE block and ECA block, our CFAM takes full account of the structure of U-Net. CFAM not only uses channel attention to adjust the channels' weights for a single feature map but also considers the interchannel relationship between the low-level and high-level features merged by the U-Net's skip connection. Studies have shown a semantic gap between two sets of features merged in U-Net's skip connections [29, 30]. The low-level features have more fine-grained information, while the high-level features have more semantic information. Convolution cannot integrate them well. To address this issue, CFAM calculates the relationship between the low-level and high-level features and adjusts their channels' weights simultaneously to help these levels of two feature maps fuse better.

CFAM uses global average pooling (GAP) and 1D convolution to capture the interchannel relationship of two sets of features to be merged in a long skip connection. Two channel attention maps are generated to refine the corresponding two sets of features before they are merged by a convolution block.

Denote one of the low-level features before downsampling in the encoder-block as *F*_*e*_ ∈ *R*^*C*×*L*×*W*×*H*^, and the corresponding high-level features after the transpose convolution in decoder-block as *F*_*d*_ ∈ *R*^*C*×*L*×*W*×*H*^, where *C*, *L*, *W*, and *H* are the number of channels, the length, the width, and the height of the feature map. First of all, we use global average pooling (GAP) to aggregate spatial information and generate the corresponding spatial statistics *s*_*e*_, *s*_*d*_ ∈ *R*^*C*^ as follows:

(2) $$\begin{array}{c} s_{e}=\text{GAP}\left(F_{e}\right)=\frac{1}{LWH}\overset{L,W,H}{\underset{i=1,j=1,k=1}{\sum }}F_{e}\left(i,j,k\right), \end{array}$$

(3) $$\begin{array}{c} s_{d}=\text{GAP}\left(F_{d}\right)=\frac{1}{LWH}\overset{L,W,H}{\underset{i=1,j=1,k=1}{\sum }}F_{d}\left(i,j,k\right). \end{array}$$

where *i*, *j*, *k* represents the voxel value at position (*i*, *j*, *k*) of a single channel in the feature map with 1 ≤ *i* ≤ *L*, 1 ≤ *j* ≤ *W*, 1 ≤ *k* ≤ *H*.

As demonstrated in [33], to capture interchannel relationships, avoiding dimensionality reduction is important, and local cross-channel interaction is helpful. So, we concatenate *s*_*e*_ and *s*_*d*_ in the channel dimension, and perform 1D convolution with kernel size *n* followed by a sigmoid activation to generate the channel attention map *M*_*e*_^*c*^(*F*_*e*_, *F*_*d*_) ∈ *R*^*c*^ for the low-level features and *M*_*d*_^*c*^(*F*_*e*_, *F*_*d*_) ∈ *R*^*c*^ for the high-level features. Finally, the refined low-level features *F*_*e*_′ ∈ *R*^*C*×*H*×*W*×*L*^ and the refined high-level features *F*_*d*_′ ∈ *R*^*C*×*H*×*W*×*L*^ can be obtained by:

(4) $$\begin{array}{c} F_{e}^{\prime }=M_{e}^{c}\left(F_{e},F_{d}\right)\cdot F_{e}=\sigma \left(f_{n}\left(s_{e},s_{d}\right)\right)\cdot F_{e}, \end{array}$$

(5) $$\begin{array}{c} F_{d}^{\prime }=M_{d}^{c}\left(F_{e},F_{d}\right)\cdot F_{d}=\sigma \left(f_{n}\left(s_{e},s_{d}\right)\right)\cdot F_{d}, \end{array}$$

where *σ* denotes the sigmoid function mapping the feature values into the range of [0, 1] and *f*_*n*_ denotes the standard 1D convolution with kernel size *n*.

### 2.6. Spatial-Wise Group Attention Module

For computer vision tasks, spatial attention is also important, so we proposed SGAM to gain spatial attention to refine the feature map in the spatial dimension. Previous works [31, 32] use average-pooling or max-pooling to aggregate channel-wise information, which cannot fully characterize the various semantic information of the feature map. The rib fracture regions are often not apparent compared with the normal rib regions and usually with various irregular shapes, so obtaining more fine-grained semantic information can enhance the CNN network's ability for feature extraction. Studies shows that group convolution can learn better feature representation than standard convolution [37]. Inspired by this, SGAM divides feature maps into several groups and simultaneously learns an attention map for each group. Each attention map focuses on a specific semantic subfeature, making SGAM to gain more fine-grained semantic information than previous works.

The detailed architecture of SGAM is illustrated in Figure 4(b). First of all, for a feature map *F* ∈ *R*^*C*×*L*×*W*×*H*^, we divide it into *G* groups along the channel dimension: *F* = {*F*_1_, ⋯, *F*_*G*_}, *F*_*i*_ ∈ *R*^*C*/*G*×*L*×*H*×*W*^. After that, for each feature group *F*_*i*_, we use 1 × 1 × 1 convolution to obtain the channel statistics *s*_*i*_ ∈ *R*^1×*L*×*W*×*H*^.

(6) $$\begin{array}{c} s_{i}=f_{1\times 1\times 1}\left(F_{i}\right), \end{array}$$

where *f*_1×1×1_ denotes a standard 3D pointwise convolution.

Then, a standard 7 × 7 × 7 convolution followed by a sigmoid activation function is performed to generate 3D spatial attention map *M*^*s*^(*F*_*i*_) ∈ *R*^1×*L*×*H*×*W*^ for each group. The final refined feature group *F*_*i*_′ ∈ *R*^*C*/*G*×*L*×*H*×*W*^ can be computed by:

(7) $$\begin{array}{c} F_{i}^{\prime }=M^{s}\left(F_{i}\right)\cdot F_{i}=\sigma \left(f_{7\times 7\times 7}\left(s_{i}\right)\right)\cdot F_{i}, \end{array}$$

where *f*_7×7×7_ denotes a standard 3D convolution with the kernel size of 7 × 7 × 7.

### 2.7. Loss Function

Since the rib fracture region is much smaller than the background, which will make the prediction of the network more biased towards the background, we use the dice loss to solve this problem. However, Dice loss is unstable in the training process, so the weighted binary cross-entropy (WBCE) loss is also introduced to address this issue.

Let *N* denote the domain of all voxels of a sample patch with length *L*, width *W*, and height *H*. $\hat{y_{i}}\in \left[0,1\right]$ is the *i*^th^ voxel of the prediction result for a sample with domain *N*, and *y*_*i*_ ∈ {0, 1} is the corresponding ground truth.

The Dice loss can be defined as:

(8) $$\begin{array}{c} L_{\text{Dice}}=1-2\frac{\sum_{i}^{N}y_{i}\hat{y_{i}}}{\sum_{i}^{N}y_{i}+\hat{y_{i}}}. \end{array}$$

The weighted BCE loss can be defined as:

(9) $$\begin{array}{c} L_{\text{BCE}}=-\frac{1}{N}\overset{N}{\underset{i=1}{\sum }}\left(\alpha y_{i}\log\left(\hat{y_{i}}\right)+\left(1-y_{i}\right)\log\left(1-\hat{y_{i}}\right)\right), \end{array}$$

where *α* is the weight of positive voxels, which is set to 5 in our experiments.

The final loss function is defined as:

(10) $$\begin{array}{c} L=L_{\text{WBCE}}+L_{\text{Dice}}. \end{array}$$

### 2.8. Implementation Details

Due to the limitation of GPU memory, the cropped 1 × 96 × 96 × 96(channel × length × width × height) 3D patches are used as the input of the network. To balance the positive and negative samples, in the training stage, 60% of the data are positive, containing at least one rib fracture, and 40% of the data are randomly sampled negative samples containing tissues without any rib fractures. Data augmentation methods including random rotation, affine, and flip are used for all samples.

In the inference stage, we use a sliding window with a window size of 96 × 96 × 96 and a step of 48 to scan the whole CT image and omit the background area without any tissues. To obtain the final result, we compute the connected component after binarizing the segmentation map using the threshold 0.4 and take the average segmentation scores of the connected component as the final detection confidence. To reduce false positives (FP), all detection proposals with volume less than 300 voxels are removed.

The CFSG U-Net is implemented in Pytorch. The kernel size *n* of CFAM in the decoder blocks is set to 5 and the group number *G* of SGAM is set to 4, which achieves the best results in our experiments. We initialize our model using the method introduced in [38] and train the model on two NVIDIA V100 32 GB GPUs with the batch size of 16 for 100 epochs. Adam optimizer with *β*_1_ = 0.9, *β*_2_ = 0.999, *ϵ* = 1 *e* − 8, an initial learning rate of 1*e* − 3, the momentum of 0.9, and weight decay of 1*e* − 4 are used for the training.

## 3. Results and Discussion

### 3.1. Results of Rib Fracture Segmentation

We first report the segmentation results of the CSFG U-Net, as shown in Figure 5; there are three true-positive results included. The ground truth is labelled by the yellow line, and the segmentation result is labelled by the red line.

Because the rib fracture area is small and narrow, and the boundary between the fracture region and the normal region is not very obvious, the dice between the segmentation result and the corresponding ground truth is not exceptionally high compared with other segmentation tasks. Due to these reasons, we did not include the quantitative segmentation result in the evaluation of our method.

### 3.2. Results of Rib Fracture Detection

As demonstrated in [26], we consider a detection is true positive if the IOU > 0.2 between any annotations. The free-response receiver-operating characteristic (FROC), which considers the sensitivity and the average number of false-positive per scan (FPs/scan), is used to evaluate the performance of models. The sensitivities are measured at five key rates, including 1/2, 1, 2, 4, and 8 FPs per scan. And the average sensitivity of these five particular rates is also used to have an overview of FROC analysis.

To verify the effectiveness of our proposed CSFG U-Net, we compare our method with several cutting-edge rib fracture detection methods proposed in recent years include FracNet [26] and VRBNet [28], which use the 3D settings. And we also compare our method with several commonly used U-Net-based deep neural networks for medical image segmentation, including 3D U-Net [39], MutiResUnet [29], Attention U-Net [40], and ResUNet [41]. Except for the differences of the CNN model, the other experimental settings of different methods are the same.

The results of the experiments are shown in Table 2. It can be seen from the results that, compared with the existing rib fracture detection models and other segmentation networks of U-Net architecture, our method achieves the highest average FPs 81.28%, which illustrates the effectiveness of our proposed network on the task of rib fracture detection.

To verify the effectiveness of the attention module we proposed, our method is also compared with several other attention modules including SE [42], CBAM [31], and ECA [43], as shown in Table 3. Here, we refer to the backbone of CFSG U-Net without CFAM and SGAM as ResUNet, which is proposed in [41]. We apply the compared attention modules in the decoder path of ResUNet as in our proposed CFSG U-Net. According to the results, the attention modules we proposed demonstrate better performance, indicating that in the U-Net architecture, our attention module can effectively help the network learn rib fracture features.

### 3.3. Ablation Studies

To justify the effectiveness of our proposed components, we conduct several ablation experiments with the leave-one-out method. The results are shown in Table 4.

To verify the effect of CFAM, we compare the performance of the whole CFSG U-Net model and the model after removing CFAM. It can be found that the model with CFAM can obtain a higher recall score, especially with low FPs/scan rates.

At the same time, to verify the effectiveness of the SGAM module, we design two experiments. In the first experiment, we remove the SGAM module from CFSG U-Net. In the second experiment, we set the number of SGAM groups to 1, equivalent to generating spatial attention without grouping. It can be seen through experiments that spatial attention can indeed improve the performance of the CNN module, and learning multiple groups of spatial attention can help the spatial attention module generate finer attention maps and reserve more fine-grained information, thereby improving the model's ability to learn rib fracture features.

## 4. Discussion

In this study, we built a deep learning model to aid in the diagnosis of rib fractures. In the experimental results, our model achieves an average sensitivity of 81.28% and a maximum sensitivity of 89.58%, which show that our method can detect rib fractures effectively and outperform the existing works. Before our work, several works used CNN to detect rib fractures but did not fully tap the potential of the CNN network. In our work, we propose a dual-attention module including CFAM and SGAM to improve the feature extraction ability of the CNN network to enhance its sensitivity and accuracy in the rib fracture detection task. We carried out several comparative and ablation experiments to test the effect of our proposed dual-attention module. Compared with other attention modules, our dual-attention module achieved the best results. At the same time, in the ablation experiments, we verified the effectiveness of CFAM and SGAM. The joint action of CFAM and SGAM improved the ability of the CNN network to detect rib fractures.

However, our work still has some limitations. First of all, our data only comes from a hospital, and the sample source is not very wide, so the model's versatility needs to be improved. In addition, in terms of data labeling, on the one hand, our data are labeled by different radiologists; it is hard to establish the labeling gold standard. On the other hand, the boundary of fractures is not obvious. These two reasons will introduce noisy labels, which may have an adverse effect on the voxel-level segmentation task. Finally, although our algorithm has obtained the highest sensitivity, it is hard to suppress false positives in a single-stage detection framework. The false-positive cases can be seen in Figures 6(a)–6(c). Several reasons cause the false positives. For instance, the rib with uneven bone mineral density can be easily misdiagnosed, and the area around the vertebra and costochondral joint might also be misdiagnosed in some CT scans.

## 5. Conclusions

In this work, to improve the ability of CNN to detect rib, we propose a novel rib fracture detection model called CFSG U-Net. Inspired by the attention mechanism of CNNs in recent years, we propose CFAM to refine features in channel perspective and SGAM to refine the semantic information in the spatial. We apply these two modules in the decoder block to reassign the weights in the channel and spatial dimensions to help the network learn rib fracture features from limited data.

To verify the effectiveness of our proposed method, we cooperated with the local hospital and established a rib fracture dataset, including 3134 rib fracture annotations for 818 CT images. And then, we conducted a series of experiments on this dataset, and the results show that the maximum sensitivity of our proposed method is 89.58%, and the average FROC score is 81.28%; these results outperformed the existing rib fracture detection system. Moreover, the ablation experiment results show that the proposed CFAM and SGAM modules surpass other attention modules in the rib fracture detection task, proving their effectiveness.

In the future, we will strengthen our work mainly from three aspects to further improve our method. Firstly, we will collect more rib fracture data and conduct multicenter research to enhance the versatility of our algorithm. In addition, we will explore how to reduce the adverse effect of noisy labels. Finally, we will continue exploring how to improve our rib fracture detection algorithm's performance in reducing false positives.

## Figures and Tables

**Figure 1:** An example of rib fracture annotation (see the red mask). (a) Axial view. (b) Coronal view. (c) Sagittal view.

**Figure 2:** The procedures of preprocessing: (a) the original CT image, (b) the binary bone region mask after thresholding at 180 HU, (c) the mask after removing small connected components, (d) the mask after morphological dilation, (e) the mask after extracting the largest connected component, (f) the extracted bone regions by applying the mask, (g) the bone regions after data normalization, and (h) the 3D view of the preprocessing output.

**Figure 3:** Our proposed CFSG U-Net. The model uses a U-Net structure consisting of four encoder blocks (E1-E4) and three decoder blocks (D1-D3). The number next to each block indicates the input size of each block. In the decoder block, *F*_*e*_ denotes the feature map from the encoder path, and *F*_*d*_ represents the feature map from the decoder path.

**Figure 4:** (a) The proposed channel-wise fuse attention module (CFAM). *F*_*e*_ denotes the feature map from the encoder path, and *F*_*d*_ denotes the feature map from the decoder path. GAP represents the global average pooling. The symbol next to the feature indicates the size of the corresponding feature. (b) The proposed spatial-wise group attention module (SGAM). *F*_*d*_ denotes the feature map from the decoder block, and the symbol in each block represents the number of channels of each block.

**Figure 5:** Three true-positive segmentation results of the CSFG U-Net. The ground truth is labelled by the yellow line, and the segmentation result is labelled by the red line.

**Figure 6:** Three false-positive cases: (a) false-positive caused by uneven bone mineral density; (b) false-positive around the vertebra area; (c) false-positive around the costochondral joint. The ground truth is labelled by the yellow line, and the segmentation result is labelled by the red line.

**Table 1:** Review of deep learning applications of rib fracture detection.

Reference	Dataset	Method used	Evaluation metrics	Research challenges
[23]	In-house dataset. No information about the dataset is mentioned in the paper	Rib region extract method and spatial coherence convolutional neural network	Accuracy, recall, and speed	There were limited comparative experiments and the potential of CNN networks was not fully researched
[24]	1,079 patients and 25,054 2D annotations from 3 different hospitals, slice thicknesses range from 1 to 5 mm	Faster R-CNN	Precision recall, and *F*1-score	This work only used 2D CNN, and no 3D information was combined. The precision and recall of this work were not particularly high
[26]	A total of 7,473 annotated traumatic rib fractures from 900 patients from a single center, slice thicknesses range from 1 to 1.25 mm	Sliding widow mechanism and a modified U-Net called FracNet	Free response receiver-operating characteristic (FROC) analysis	This article only carried out a single-center study, and the landscape of deep neural networks was not fully explored
[28]	8,529 chest CT images and 33,828 annotations, slice thickness of CT images was 0.625 mm	Rib fracture detection pipeline consisting of five stages: rib segmentation, vertebra detection, rib labeling, rib fracture detection, and rib fracture classification. VRB-Net for rib fracture detection	Recall, precision, and *F*1 score	The ground truth for detection and classification may include incorrect cases caused by incorrect annotation

**Table 2:** Comparison experiment results of our proposed method, several cutting-edge rib fracture detection methods, and commonly used U-Net architecture deep neural networks are included. The best results are marked in bold. FPs/scan denote false positives per scan.

Methods	Sensitivities (FPs/scan)					
	0.5	1	2	4	8	Avg.
CFSG U-Net	67.15	76.92	**84.78**	**87.98**	**89.58**	**81.28**
FracNet	60.10	70.03	79.01	82.21	85.90	75.45
VRBNet	**71.31**	**77.56**	82.21	85.25	85.25	80.32
3D U-Net	59.46	69.23	77.72	81.73	85.26	74.68
MutiResUnet	61.70	71.79	80.93	83.81	87.18	77.08
Attention U-Net	61.54	72.12	81.09	84.29	87.34	77.28
ResUNet	60.90	70.99	80.13	83.33	86.70	76.41

**Table 3:** Comparison experiment results of different attention methods. The best results are marked in bold. ResUNet denotes the backbone proposed in [41].

Methods	Sensitivities (FPs/scan)					
	0.5	1	2	4	8	Avg.
CFSG U-Net	**67.15**	**76.92**	**84.78**	**87.98**	**89.58**	**81.28**
ResUNet+CBAM	65.22	75.48	83.49	86.70	88.94	79.97
ResUNet+ECA	62.66	73.08	81.41	84.78	87.98	77.98
ResUNet+SE	63.14	73.72	81.73	85.10	87.98	78.33

**Table 4:** Ablation experiment results for our proposed method. The best results are marked in bold. w/o denotes “without,” w/ denotes “with.” *G* denotes the number of groups of SGAM.

Methods	Sensitivities (FPs/scan)					
	0.5	1	2	4	8	Avg.
CFSG U-Net	**67.15**	**76.92**	**84.78**	**87.98**	**89.58**	**81.28**
w/o CFAM	62.18	72.76	81.41	84.46	87.50	77.66
w/o SGAM	64.10	74.52	82.53	85.74	88.46	79.07
w/ SGAM *G* = 1	66.35	76.28	84.13	87.50	89.26	80.71

## Data Availability

The data used to support the findings of this study are available from the corresponding author upon request.
